This article has been retracted.

# A Retrospective Analysis of 1,595 Cases: Comparing the Characteristics of Total Knee Arthroplasty between Tibetans Living in the Plateau and Han of the Sichuan Basin

**DOI:** 10.1155/2022/5331346

**Published:** 2022-04-04

**Authors:** Jing Guo, Qiang Xu, Menghui Gao, Qingyan Zhang

**Affiliations:** Lower Limb Department, Sichuan Province Orthopedic Hospital, Chengdu, Sichuan 610041, China

## Abstract

**Background:**

Total knee arthroplasty is an effective treatment for end-stage knee arthritis. Studies' date have shown that the demand for knee replacements continues to increase worldwide. Although racial disparities have been previously reported in the utilization of total knee arthroplasty in western countries, however, there are few similar studies in China.

**Objectives:**

Retrospective analysis of medical records identified the characteristics of Tibetan patients who had undergone total knee arthroplasty living in plateau and their differences with Hans living in Sichuan Basin.

**Methods:**

The patients with unilateral primary total knee arthroplasty in Sichuan Orthopedic Hospital from 2015 to 2020 were enrolled. Analyze and compare the demographic characteristics (age, body mass index, and occupation) and pathogenesis characteristics (disease duration, exacerbation period, treatment methods, etc.) of the plateau Tibetans and the Hans of the Sichuan Basin.

**Results:**

1595 eligible patients were reviewed, including 541 Tibetan patients and 1054 Han patients, The average age of Tibetan patients was lower than that of Han patients (*P* < 0.001); the average BMI index of Tibetan patients was higher than that of Han patients (*P* < 0.001). And obese people account for more; the occupational distribution of Tibetan patients is more concentrated, mainly farmers. Tibetan patients have a longer course of disease than Han patients (*P* < 0.001).

**Conclusions:**

The social background and geographical environment of the Tibetan population are different from those of the Han. Tibetans living on plateaus have an earlier illness, a longer course of illness, a more obvious trend of younger, age and fewer opportunities for regular treatment during the illness.

## 1. Introduction

Total knee arthroplasty (TKA) is an effective treatment for end-stage knee osteoarthritis (KOA) [1] that can significantly improve the quality of life of patients. Recently, the number of TKA procedures has continued to increase around the world. In Italy, the number of TKA increased by 262% from 2001 to 2016 [2], and in the United States, the number increased by 210% from 2010 to 2020 [3]. The number of TKA procedures in European and American countries is predicted to continue to increase [4–8]. Around 50,000-70,000 patients undergo TKA in China every year [9]. Developed countries in Europe and America have carried out extensive epidemiological research on TKA patients of different races and geographical regions that have improved the diagnosis and treatment of TKA [10]. However, the characteristics of multiethnic TKA patients in China have not been analyzed, particularly in the Tibetan population living on plateaus. This study involved a retrospective analysis of the TKA procedures carried out at the Sichuan Province Orthopedic Hospital from 2015 to 2020 and compared the epidemiological characteristics of TKA between the Tibetan and Han populations. These data were used to inform the improved diagnosis and treatment of Tibetan TKA patients, promote the fair and reasonable distribution of care resources, and improve the life quality and health level of Tibetan people.

## 2. Method

### 2.1. Study Date and Site

Patient medical records were collected from the Sichuan Province Orthopedic Hospital from January 1, 2015 to December 31, 2020.

### 2.2. Objects of Study

This study involved a total of 1,595 patients who underwent the unilateral primary TKA from the Tibetan population living on the plateau at an average altitude of >1500 m and from the Han population in the Sichuan Basin. The total study population included 541 Tibetan patients (180 males and 361 females) and 1,054 Han patients (225 males and 829 females).

### 2.3. Inclusion Criteria

Patients newly diagnosed with knee osteoarthritis were included in this study.

### 2.4. Exclusion Criteria

Patients with knee-joint repair, nonosteoarthritis and unclassified arthritis, non-Han and Tibetan patients, and plateau migrants were excluded from the study.

### 2.5. Primary Observation Index

#### 2.5.1. The Demographic Characteristic Index for the Tibetan and Han Populations

*(1) Age*. The patients were divided into 5 age groups as follows: <49 years, 50-59 years, 60-69 years, 70-79 years, and ≥80 years of age.

*(2) Body Mass Index (BMI)*. According to *the Guidelines for Prevention and Control of Overweight and Obesity in Chinese Adults* (2006), the BMIs of the patients were divided into four groups as follows, <18.5 (low weight), 18.5 to 23.9 (normal weight), 24 to 27.9 (overweight), and ≥28 (obesity).

*(3) Occupation*. According to the *Classification of Physical Labor Intensity* (2007), the occupational labor intensity of the patients was divided into light, medium, heavy labor, and extremely heavy labor. The occupations of the patients were classified according to labor intensity, labor time, work posture, and other factors. The work performed by farmers and porters was defined as extremely heavy labor, the work of sales personnel was defined as heavy labor, the work done by workers is defined as medium labor, and the work of public security personnel, teachers, cadres, and retirees was defined as light labor.

#### 2.5.2. Characteristic Indices of Illness in the Tibetan and Han Patients

*(1) Disease Course*. According to the *Expert Consensus on the Phased Treatment of Knee Osteoarthritis* (2018), the KOA disease course was divided into the initial, early, middle, and late stages. To facilitate comparative analysis, the disease course was defined as the illness and exacerbation periods. The illness period included the initial, early, and middle stages with a Visual Analogue Scale (VAS) ranging from 0 to 4 points and X-ray radiography conforming to the Kellgren-Lawrence (K-L) grades [11] I-III. The exacerbation period included the late stage with a VAS ranging from 4 to 10 points and K-L Grade IV.

*(2) Treatment during Illness*. In this study, the treatment measures during the illness were divided into standard and nonstandard treatments. The standard treatment referred to the periodic and individualized treatment measures recommended in *the Guidelines for Diagnosis and Treatment of Osteoarthritis* (2018). The nonstandard treatment referred to untreated and self-medication measures.

### 2.6. Statistical Methods

SPSS 25.0 software was used for statistical analysis. The count data is represented as the count and percentage (*n*, %). Due to the large sample size, a Pearson-*x*^2^ test was used for the comparison between the groups and the measurement data is expressed as the mean ± standard deviation(*x* ± *s*). A *t*-test was used for comparison between the groups. A tank sum test was used to compare data that were not normally distributed. The level of statistical significance was set as *α* equal to 0.05. Differences were considered statistically significant when the 2-tailed test *P* value was <0.05.

## 3. Results

### 3.1. Age

The average age of the Tibetan patients undergoing TKA was 62.37 ± 7.63 years, and the average age of the Han patients undergoing TKA was 67.74 ± 7.79 years. The data show that the average age of the Tibetan patients was significantly lower than the Han patients (*t* = 13.11, *P* < 0.0001 (Table 1). The proportions of Tibetan patients under the age of 49, between 50 and 59 years old, and between 60 and 69 years old, were significantly higher than the Han patients in the same age groups (*x*^2^ = 127.90, *P* < 0.0001) (Table 2). Tibetan patients undergoing TKA showed an overall younger trend during 2015 and 2020 that decreased from 63.5 years old to 60.52 years old. The average age of the Han patients did not change significantly with an average between 67 and 68 years (Table 3, Figure 1).

### 3.2. Gender

A total of 405 male patients and 1,190 female patients were included in the study resulting in an overall male to female ratio of 1 : 2.94. The male to female ratio was significantly different between the groups at 1 : 2.01 in the Tibetan patients and 1 : 3.68 in the Han patients (*x*^2^ = 26.83, *P* < 0.0001) (Table 4). By comparing with gender over time, no significant change in the proportion of male Tibetan and Han patients (*P* > 0.05) was observed. The proportion of female Tibetan patients showed an increasing year-on-year trend, and the proportion of female Han patients showed little change, and the difference was statistically significant (*x*^2^ = 39.89, *P* < 0.0001) (Table 5, Figure 2).

### 3.3. BMI Characteristics

The average BMI was significantly higher in the Tibetan patients (26.94 ± 4.05) than the Han patients (25.49 ± 3.38) (*t* = 7.16, *P* < 0.0001) (Table 6). Due to differences in the distribution of BMI between the populations, the proportion of Tibetan patients that were obese (39.6%) was significantly higher than the proportion of overweight Han patients (46.2%) (Figure 3) (*χ*^2^ = 52.99, *P* < 0.0001) (Table 7). Comparison of the Tibetan and Han population based on gender factors showed that the difference in average BMI was not statistically significant (*P* > 0.05) (Table 8).

### 3.4. Occupation

A significant difference in the occupational distribution was observed between the Tibetan and Han patients significant (*χ*^2^ = 16.302, *P* = 0.0002) (Table 9). According to the comparative analysis of labor intensity, our data showed that the proportion of Tibetan patients in the light and heavy labor groups was significantly higher than the Han patients with a bipolar distribution (*χ*^2^ = 16.302, *P* = 0.0009) (Table 10).

### 3.5. Disease Course

The average duration of the disease in the Tibetan patients (10.12 ± 6.93 years) was significantly longer in the Han patients (9.05 ± 7.42 years). Also, the average exacerbation duration in the Tibetan patients (2.16 ± 2.41 years) was significantly longer than the Han patients (1.50 ± 1.89 years) (*Z*^1^ = 5.65, *Z*^2^ = 6.44, P1, *P*^2^ < 0.0001) (Table 11).

### 3.6. Treatment Methods

The proportion of Tibetan patients who received standard treatment during the whole course of the disease was significantly lower than the Han patients (*x*^2^ = 73.38, *P* < 0.0001) (Table 12).

## 4. Conclusion

### 4.1. Tibetan Patients Treated with TKA Were Significantly Younger than Han Patients

The average age of the Tibetan patients treated with TKA was 62.37 ± 7.63 which was lower than the Han patients (67.74 ± 7.79 years). The average period of the disease course and aggravation in the Tibetan patients was 1.07 and 0.66 years, respectively, which were longer than the Han patients. Based on these data, we hypothesized that the age of onset of osteoarthritis (OA) in Tibetan patients was younger than in Han patients. Studies have shown that the incidence of OA in the plateau and alpine areas is higher than in plain areas [12].

The pathogenesis of OA may be related to hypoxia-inducible factors (HIFs) [13] and cold stimulation. HIF-2*α* is a catabolic regulator that can degrade articular cartilage [14]. HIF-2*α* can also promote cartilage ossification by inducing hypertrophic differentiation in chondrocytes [15]. HIF-2*α* is expressed at high levels in a mouse model of cartilage degradation in the articular cartilage of OA patients [16]. Cold stimulation can lead to imbalances in the microenvironment of joint tissues and increase the expression of inflammatory factors. It can also activate the cold-sensitive ion channels TRPA1 and TRPM8 which are members of the transient receptor potential (TRP) family [17]. Finally, it can promote the overexpression of matrix metalloproteinases (MMPs) [18] and enhance the destruction of cartilage.

Based on these findings, the synergistic effect of low temperature and cold factors may be the main reason for the earlier onset of OA and the younger age of TKA in Tibetan patients compared to Han patients. In this study, we also found a younger trend of Tibetan who received TKA. This may be due to transportation in the Tibetan area being increasingly convenient. Also, the difficulty and cost of transportation to the mainland for medical treatment are reducing and so middle-aged Tibetan patients with OA have increasing access to treatment.

### 4.2. The Proportion of Tibetan Female Patients Receiving TKA Is Significantly Lower than Han Patients but Continues to Increase Year by Year

Gender is the main risk factor associated with OA [19]. It has been reported that the incidence rate of postmenopausal women is about 3 times that of men in the same age group [20]. Under the same imaging indications, female patients have more serious clinical symptoms [21] that are related to decreased estrogen levels. Estrogen can regulate the balance between cartilage decomposition and synthesis by affecting the expression of MMPs to protect chondrocytes [22, 23]. In this study, the male to female ratio of Han patients was 1 : 3.68 which was consistent with the results of a previous study [24]. In the gender analysis of the Tibetan patients, considering that Tibetan women are also affected by hypoxia and cold at high altitudes, we predicted that the proportion of male and female patients should be higher than the Han patients. However, the ratio of males to female patients was only 1 : 2.01 which was lower than expected. We hypothesize that most Tibetan women have a low level of education and cannot communicate effectively in Chinese Communication [25], and so they do not seek treatment without permission after an illness. Also, Tibetan women usually have no dominant position in family economic life, and so after they get sick they rarely receive treatment and the motivation to obtain treatment intention. Recently, our hospital and the major hospitals in the province have actively carried out medical development in the poor Tibetan areas of Western China. Many doctors are trained in Ganzi, Aba prefecture and Muli Tibetan to perform effective TKA, and inform the Tibetan people of the treatment. During this study, the proportion of Tibetan female patients in our hospital increased year on year to reflect the sustainable development of medical technology in Tibetan areas.

### 4.3. Tibetan Patients Have a Higher BMI and a Higher Proportion of Patients Are Obese

Obesity is an important risk factor in the pathogenesis of OA [26], because heavier inflict more serious wear on articular cartilage [27]. The excessive accumulation of fat can also interfere with the growth and repair of cartilage [28], acting to accelerate degenerative changes in bones and joints. In this study, the average BMI of the Tibetan patients was 1.45 times higher than the Han patients. These observations may be related to the diet structure of Tibetans as they usually prefer to eat beef, mutton, and less healthy foodstuffs. Also, there were no gender differences in BMI observed in this study; however, other studies have reported that the impact of high BMI is greater in women than in men [29] yet the mechanism remains to be fully determined. Further multicenter studies in large sample cohorts are required to investigate the underlying basis of these data.

### 4.4. The Occupational Distribution of Tibetan Patients Is Much more Concentrated than That of Han Patients

We found that Tibetan and Han patients treated with TKA mainly include members of the population who engage in heavy or extremely heavy labor which is consistent with other studies [30]. We speculated that the mechanistic basis of these observations may be the acceleration of knee wear or the aggravation of OA due to an increased knee load. The Tibetan patients are mainly farmers whilst the Han patients have more varied occupations such as sales people. Most of the sick workers were male who engaged in machinery manufacturing and were required to bend their knees for long periods. Also, the patients who were sales staff were mainly women who were required to stand for long periods. Therefore, in daily life, individuals should avoid long-time standing, knee bending, and weight-bearing exercises. Health education should also be carried out amongst all ethnic groups to strengthen the awareness of rational and healthy knee use.

### 4.5. Tibetan Patients Received less Standard Treatment than Han Patients

In this study, we collected and analyzed the clinical information of Tibetan and Han patients during the treatment of TKA. The number of Tibetan patients that received nonstandard treatment before attending hospital was higher than Han patients. These data may be due to economic restrictions, religious beliefs, and differences in culture and customs. We found that Tibetan people generally lack awareness of self-care. Also, the medical conditions in Tibetan areas are relatively underdeveloped. Most patients do not receive standard treatment at the early stages of the disease and often choose to go to temples for divination or use nonprescribed drugs rather than attend hospitals.

The special ecological environment, lifestyle, cultural background, demographics, and disease characteristics of Tibetan TKA patients in the plateau region are significantly different from Han patients in the Sichuan basin. In this study, the characteristics of Tibetan TKA patients who had been living on the plateau for a long time were identified by retrospective analysis of medical records. However, as this study was conducted as a single-center investigation and the sample size was restricted, there may be some biases. To improve the health of Tibetan people, further multicenter studies are required in Tibetan TKA patients.

## Figures and Tables

**Figure 1:** The age trends of the Tibetan and Han patients.

**Figure 2:** Trends of morbidity in the female Tibetan and Han patients.

**Figure 3:** BMI distributions in the Tibetan and Han patients.

**Table 1:** Comparison of the average ages of Tibetan and Han patients (*n*, $\bar{x}\pm s$).

Ethic group	Number of cases *N*	Average age $\bar{x}\pm s$	Minimum age	Maximum age	Difference of average age	*t*	*P*
Han	1054	67.74 ± 7.79	42	93	5.37	13.11	<0.0001
Tibetan	541	62.37 ± 7.63	36	92			

**Table 2:** Age distribution of the Tibetan and Han patients (*n*, %).

Age group	Number of cases *n*	Tibetan (*n*, intragroup %)	Han (*n*, intragroup %)	*x* ^2^	*P*
49 years old and below	40	28 (5.18%)	12 (1.14%)	127.90	<0.0001
50-59 years old	283	151 (27.91%)	132 (12.52%)		
60-69 years old	701	252 (46.58%)	449 (42.6%)		
70-79 years old	506	101 (18.67%)	405 (38.43%)		
80 years old and above	65	9 (1.66%)	56 (5.31%)		

**Table 3:** Analysis of the average age and time trend for the Tibetan and Han patients ($\bar{x}\pm s$).

Ethnic group	2015	2016	2017	2018	2019	2020
Tibetan	63.48 ± 8.25	63.32 ± 9.65	63.82 ± 9.24	62.83 ± 7.17	61.32 ± 5.68	60.51 ± 5.87
Han	66.49 ± 8.39	67.94 ± 7.88	67.65 ± 7.71	67.40 ± 7.46	68.49 ± 7.71	67.43 ± 7.68

**Table 4:** Summary of the gender distributions of the Tibetan and Han patients (*n*, %).

Ethnic group	Tibetan	Han	Total	*x* ^2^	*P*
*Gender*					
Male (*n*, %)	180 (33.3%)	225 (21.3%)	405	26.83	<0.0001
Female (*n*, %)	361 (66.7%)	829 (78.7%)	1190		
Proportion (male: female)	1 : 2.01	1 : 3.68	1 : 2.94		
Total (*n*, %)	541 (100%)	1054 (100%)	1595		

**Table 5:** Comparison of gender and time distribution of the Tibetan and Han patients (*n*, %).

Ethnic group	Time grouping						Total	*χ* ^2^	*P*
	2015	2016	2017	2018	2019	2020			
Tibetan male	9	30	40	28	51	22	180		
*n*, (% of Tibetan)	(39.13%)	(37.97%)	(34.78%)	(31.82%)	(30.56%)	(32.3%)	(33.27%)	10.16	0.071
Han male	23	55	42	29	46	30	225		
*n*, (% of Hans)	(21.7%)	(20.68%)	(23.73%)	(21.01%)	(19.25%)	(23.44%)	(21.35%)		
Tibetan female	14	49	75	60	113	50	361		
*n*, (% of Tibetan)	(60.87%)	(62.03%)	(65.22%)	(68.18%)	(69.44%)	(67.7%)	(66.73%)	39.98	<0.0001
Han female	83	211	135	109	193	98	829		
*n*, (% of Hans)	(78.30%)	(79.32%)	(76.27%)	(78.99%)	(80.75%)	(76.56%)	(78.65%)		

**Table 6:** Comparison of the average BMI values between the Tibetan and Hans populations ($\bar{Χ}\pm \text{s }$).

Ethnic group	Tibetan	Han	Average difference	*t*	*P*
BMI index	26.94 ± 4.05	25.49 ± 3.38	1.45	7.16	<0.0001

**Table 7:** The distribution of BMI in the Tibetan and Han patients (n, %).

Ethnic group	BMI distribution					
	<18.5	18. 5-23. 9	24-27.9	≥28	*χ* ^2^	*P*
	Light weight	Normal weight	Overweight	Obesity		
Tibetan	5 (0.9%)	110 (20.3%)	212 (39.2%)	214 (39.6%)	52.99	<0.0001
Han	15 (1.4%)	314 (29.8%)	486 (46.2%)	238 (22.6%)		
Total	20	424	698	452		

**Table 8:** Comparison of gender and BMI between the Tibetan and Han patients ($\bar{Χ}\pm s$).

Ethnic group	Gender			
	Male	Female	*t*	*P*
Tibetan	26.65 ± 3.46	27.09 ± 4.32	1.28	0.203
Han	25.25 ± 3.42	25.55 ± 3.36	1.18	0.237

**Table 9:** The occupational statistics of the Tibetan and Han patients (*n*, %).

Ethnic group	Occupation										
	Cadre	Worker	Public security personnel	Teacher	Doctor	Farmer	Porter	Retiree	Shop employee	*χ* ^2^	*P*
Tibetan	47	28	0	1	1	357	9	34	64	36.26	0.0002
	(8.7%)	(5.2%)	(0%)	(0.2%)	(0.2%)	(66%)	(1.7%)	(6.3%)	(11.8%)		
Han	35	101	1	4	2	648	34	82	147		
	(3.3%)	(9.6%)	(0.1%)	(0.4%)	(0.2%)	(61.5%)	(3.2%)	(7.8%)	(13.9%)		
Total	82	129	1	5	3	1005	43	116	211		
	(5.1%)	(8.1%)	(0.1%)	(0.3%)	(0.2%)	(63%)	(2.7%)	(7.3%)	(13.2%)		

**Table 10:** The occupation distribution of the Tibetan and Han patients (*n*, %).

Ethnic group	Labor intensity					
	Light labor	Medium labor	Heavy labor	Extremely heavy labor	*χ* ^2^	*P*
Tibetan	83 (15.3%)	28 (5.2%)	73 (13.5%)	357 (66%)	16.30	0.0009
Han	124 (11.8%)	101 (9.6%)	181 (17.2%)	648 (61.5%)		
Total	207	129	254	1005		

**Table 11:** Comparison of the disease prevalence and exacerbation period between the Tibetan and the Han patients (*x* ± *s*).

Ethnic group	Number of cases (*n*)	Average duration of disease (year)	Average exacerbation duration of disease (year)
Han	1054	9.05 ± 7.42	1.50 ± 1.89
Tibetan	541	10.12 ± 6.93	2.16 ± 2.41
*Z*		5.646	6.437
*P* (2-tailed)		<0.0001	<0.0001

**Table 12:** Comparison of the treatment methods between the Tibetan and the Han patients (*n*, %).

Ethnic group	Treatment method			
	Nonstandard treatment	Standard treatment	*X* ^2^	*P*
Tibetan	381 (70.4%)	160 (29.6%)	73.38	<0.0001
Han	505 (47.9%)	549 (52.1%)		
Total	886 (55.5%)	709 (44.5%)		

## Data Availability

The labeled dataset used to support the findings of this study is available from the corresponding author upon request.
